# Interpretation of Electrocardiogram Heartbeat by CNN and GRU

**DOI:** 10.1155/2021/6534942

**Published:** 2021-08-29

**Authors:** Guoliang Yao, Xiaobo Mao, Nan Li, Huaxing Xu, Xiangyang Xu, Yi Jiao, Jinhong Ni

**Affiliations:** School of Electrical Engineering, Zhengzhou University, Zhengzhou 450001, China

## Abstract

The diagnosis of electrocardiogram (ECG) is extremely onerous and inefficient, so it is necessary to use a computer-aided diagnosis of ECG signals. However, it is still a challenging problem to design high-accuracy ECG algorithms suitable for the medical field. In this paper, a classification method is proposed to classify ECG signals. Firstly, wavelet transform is used to denoise the original data, and data enhancement technology is used to overcome the problem of an unbalanced dataset. Secondly, an integrated convolutional neural network (CNN) and gated recurrent unit (GRU) classifier is proposed. The proposed network consists of a convolution layer, followed by 6 local feature extraction modules (LFEM), a GRU, and a Dense layer and a Softmax layer. Finally, the processed data were input into the CNN-GRU network into five categories: nonectopic beats, supraventricular ectopic beats, ventricular ectopic beats, fusion beats, and unknown beats. The MIT-BIH arrhythmia database was used to evaluate the approach, and the average sensitivity, accuracy, and F1-score of the network for 5 types of ECG were 99.33%, 99.61%, and 99.42%. The evaluation criteria of the proposed method are superior to other state-of-the-art methods, and this model can be applied to wearable devices to achieve high-precision monitoring of ECG.

## 1. Introduction

Heart-related diseases have become the world's leading cause of death, according to the World Health Organization (WHO) [1]. Today, the most effective way to diagnose heart disease is to take a patient's electrocardiogram, which can be read by a doctor to determine if the patient has a heart-related disease. The process of reading an ECG is time-consuming and laborious and depends on the subjective judgment of the doctor. In recent years, the number of people diagnosed with electrocardiogram (ECG) has increased year by year, as has the number of ECGs that need to be interpreted. However, there are only a limited number of doctors who can read the ECG images. Therefore, it is urgent to develop an accurate and efficient ECG diagnosis algorithm [2].

At present, most cutting-edge algorithms for this problem divide the MIT-BIH arrhythmia database into 5 categories according to the American Association for the Advancement of Medical Devices (AAMI) standard: nonectopic beats (N), supraventricular ectopic beats (S), ventricular ectopic beats (V), fusion beats (F), and unknown beats (Q) [3]. Many classification algorithms have been designed to classify ECG signals according to these five categories. In recent decades, machine learning algorithms have made great achievements in the field of ECG classification, such as random forest [4], rough set theory [5], support vector machines [6, 7], and neural network [8, 9]. Among many machine learning algorithms, the convolutional neural network (CNN) algorithm of convolutional neural network has strong feature extraction and self-learning ability. Compared with traditional methods, the CNN algorithm has better classification performance and does not need feature extraction. It can directly classify the original ECG signals and eliminate human interference.

Recently, many CNN-related methods have achieved good results in solving the problem of ECG detection. Jun et al. converted 1D ECG data into 2D grayer images and proposed to use the 2DCNN classifier to obtain features of more ECG signals, which requires much more computational effort than the use of the 1D neural network [10]. Acharya et al. used data enhancement technology to obtain a balanced dataset and trained CNN with enhanced data. Their classifier only used simple convolution operation and the accumulation of subsamples to construct CNN [11]. Hannun et al. designed 1DCNN with a residual structure, which did have advantages in training efficiency, but did not extract the long-term dependence contained in ECG sequences [12]. Ihsanto et al. used a neural network to realize the 19 classifications of ECG signals [13].

Although the existing research methods have good performance, they still have the following defects: (1) Most of the methods simply deepen the number of network layers without other improvements. (2) The problem of accuracy distortion caused by an unbalanced dataset is not solved. (3) In many methods, the original signal is directly input into the classifier, and the noise part of the signal will interfere with the final classification effect. (4) Many algorithms simply pick out certain categories in the dataset for classification, and there is no specific standard for unified classification, so it is difficult to compare the performance of various algorithms.

In addition, it should be noted that ECG signals reflect the time series of cardiac activity through a series of complex mapping relations. Although the classification effect of CNN is very good, it lays more emphasis on the calculation of spatial structure, so it is more suitable for spatial data such as pictures, while the recurrent neural network (RNN) can extract the time characteristics in time series. In recent years, RNN have achieved success in several applications involving sequential or temporal data. For example, it has been widely used in speech recognition, natural language processing, machine translation, and other fields. The gated recurrent unit (GRU), as a new type of RNN, shows good performance in long sequence applications. It can achieve a better feature extraction effect in the case of saving computation and is very suitable for such a long time series of ECG signals. Considering such factors, a new classifier combining CNN and GRU was proposed, and a good classification effect was achieved on the MIT-BIH arrhythmia database.

Although the knowledge of ECG interpretation continues to evolve, automatic classification of ECG remains a significant challenge due to the need for high safety in the medical field and the diversity and variability of ECG types. In this study, the goal is to design an ECG classifier with high accuracy for the above problems. Firstly, a preprocessing scheme is designed for denoising and equalization of ECG data. Then, a new deep learning classifier is proposed by combining GRU and CNN technologies. Finally, the performance of the model is verified by using the MIT-BIH database. The proposed method uses shallow layer networks to achieve excellent classification results.

The main contributions of this work are the following:

1. By using the prior knowledge of frequency domain and time domain of ECG data, the idea of using the CNN structure to extract data features and using the GRU structure to extract data time features is proposed
2. A featureless lightweight convolutional neural network is designed to represent and recognize ECG signals. The CNN model can well explore the waveform features, morphological characteristics, and time domain features of ECG signals, by the combination of convolution blocks and gate recurrent unit (GRU)
3. The well-known MIT-BIH arrhythmia database was used to validate the model performance and compare the experimental results with the scientific literature reviewed. The results show that the proposed model is more efficient than the current technology in terms of accuracy

The remainder of this paper is organized as follows. In Section 2, the methods designed and the techniques used are described. Experiments, evaluation, and result comparison are presented in Section 3. The conclusion is given in Section 4.

## 2. Materials and Methods

In this part, the datasets used in the study and the data processing steps are first introduced, and then, the proposed CNN model and the selection of optimizer activation functions used in the proposed method are described.

### 2.1. Data Description

For this experiment, the MIT-BIH arrhythmia database was used to verify the performance of the proposed model [15] (the MIT-BIH arrhythmia database can be downloaded from https://physionet.org/content/mitdb/1.0.0/https://physionet.org/content/mitdb/1.0.0/). The database consisted of 48 sets of ECG signals from 47 patients in the arrhythmia laboratory, with a duration of 30 minutes, and each signal is then digitized at 360 Hz. The ECG signal from the MIT-BIH database consists of a “.HEA” text header file, a “.DAT” binary data file, and an “.ATR” annotation file in which the ECG specialist records the diagnostic information of the corresponding ECG signal. The header file specifies detailed information, including sample number, sampling frequency, ECG signal format, type of ECG conductance, patient history, and detailed clinical information. In binary files, the signal is stored in 212 format and binary comment files consist of beat comments [15, 16]. The WFDB-Python tool is used to read the ECG data into an array based on the contents of the annotated file. In our experiments, only data from the MLII lead were used. Based on the information available in the database, the signal is segmented into heartbeats centered on each R peak, and its corresponding type is recorded. Each heartbeat consisted of 186 sample points (85 samples before R peak and 100 samples after R peak). The AAMI standard is used to classify the MIT-BIH dataset, and the specific description of this standard can be seen in Rajesh and Dhuli's [14] study. According to AAMI recommendations, 109,446 ECG signals are classified into five categories, as shown in Table 1.

### 2.2. Preprocessing

To achieve the optimal performance of the proposed model, the original data need to be preprocessed first. The data preprocessing part mainly includes the following four steps.

#### 2.2.1. Wavelet Denoising

Noise in the ECG signal includes human EMG signals, electrical noise signals of acquisition equipment, and baseline drift [17]. Wavelet transform can decompose the signal containing noise into the basis function of time and scale, so it can achieve better denoising effect while retaining the edge and details of the original signal [18, 19]. The original signal was decomposed into 9 wavelet components by wavelet 6 (db6). Wavelet components of levels 3-9 are used to reconstruct the signal. The signal before and after denoising is shown in Figure 1.

#### 2.2.2. Heartbeat Signal Extraction

Each beat is extracted according to the R peak position marked by the annotation file in the MIT-BIH database. Each beat signal is composed of 85 sampling points before the annotation position and 100 sampling points after the annotation position.

#### 2.2.3. Normalization

The value range of each sampling point of the ECG signal is normalized to between 0 and 1. Normalizing the initial input of the model can improve the convergence speed in the process of model training, and its essence is to speed up the calculation speed of gradient descent. At the same time, the normalization process makes the data between different dimensions have better comparison, so normalization has the benefit of improving the accuracy of the model [20].

#### 2.2.4. Data Augmentation

Large and balanced datasets are the guarantee for training excellent models [21]. However, in the MIT-BIH database, the number of category N ECG signals is far greater than that of category F ECG signals. If such a dataset is directly used to train the model, the model will tend to predict the sample as the category with a large number of samples. Therefore, resampling, scaling, clipping, and other operations are used for data enhancement of S, V, Q, and F, while N types of data are randomly selected so as to be similar to the number of other types of data [22].

The following methods are used for data augmentation.

*Resampling*: the original data is subsampled and zeroed at the end of the data to make it the same length as the original data.

*Scaling*: the mean value of two adjacent data points was inserted between each two adjacent data points, the length of the data was expanded, and then, the obtained data was cropped to make its length the same as the original data.

*Clipping*: some data from both sides of the data were randomly deleted and the cropped part with zeros was supplemented.

### 2.3. Architecture of Proposed Model

After the preprocessing is completed, this part introduces the network model and its design ideas. Generally speaking, there are two main criteria for detecting abnormal ECG signals: abnormal ECG pulse shape and the difference in the occurrence time of abnormal ECG fluctuations. If a model can handle the above two conditions, it needs (1) good feature extraction ability to reconstruct as many ECG waveforms as possible and (2) the ability to analyze time series data. In the field of deep learning, there are two widely used networks, namely, CNN and GRU. CNN focuses on feature extraction, and GRU focuses on time series analysis [23]. Existing good studies either use stacked GRU or use deep CNN alone for electrocardiogram classification. However, we have discovered that when designing ECG classifiers based on GRU alone, learning the local features of the input data will become a huge challenge and ultimately an almost infinite training time. On the other hand, a single CNN structure can effectively extract the local features of data. However, CNN was originally used to classify data that did not include time information such as images, and the single CNN structure would lose the time information of the data. Therefore, it is natural for us to consider combining CNN and GRU to solve the problem of electrocardiogram classification.

#### 2.3.1. Architecture Overview

Based on the previous analysis of the characteristics of ECG signals and CNN, a deep learning algorithm framework is proposed, as shown in Figure 2, which is used to extract and classify ECG signals and is mainly composed of CNN and GRU. Firstly, the original data was automatically extracted by CNN, and then, the extracted sequence features were input into GRU to extract time-dependent characteristics. Finally, the Dense layer and Softmax layer were used to classify the ECG signals.

#### 2.3.2. Description of the CNN Module

The proposed CNN model structure is shown in Figure 2. Considering that ECG signals in the MIT-BIH dataset are all time series, the one-dimensional convolutional neural network can best extract the features of the original signals. Therefore, the one-dimensional CNN model is used to carry out a one-dimensional convolution layer and filter on the input data. First, a convolutional layer is used to propose preliminary features of the original data, and then, a feature extraction module composed of two convolutional layers, a batch normalization (BN) operation, a rectified linear unit (ReLU), and a pooling layer is used to extract deeper features of ECG signals. Six feature extraction modules are superimposed to form the backbone of the model, which achieves the best classification effect. Adding ReLU and BN to each LFEM can add nonlinear factors in the operation process and improve the training speed [24]. The convolution layer extracts the local features of the data through the convolution operation [25]. The process of the convolution layer can be described by

(1) $$\begin{array}{c} x_{k}^{l}=f\left(\underset{i\in M_{k}}{\sum }\;x_{i}^{l-1}\cdot \omega_{ik}+b_{k}\right), \end{array}$$

where *M*_*k*_ is the effective range of the convolution kernel, *x*_*k*_^*l*^ represents the output of the *k*th neuron in layer *l*, *b*_*k*_ represents the bias of the *k*th neuron in layer *l*, *ω*_*ik*_ represents the convolution kernel between the *i*th neurons in layer *l* and the *k*th neurons in layer *l* − 1, and *f*(·) represents the ReLU activation function.

The subsampling layer can reduce the computation while ensuring the extraction of good features in the training process [26]. Max-pooling is adopted to obtain the maximum value in the data neighborhood to replace the features of the network of the upper layer. The operation process is shown in

(2) $$\begin{array}{c} x_{k}^{l}=\text{subsample}\left(x_{k_{\text{cluster}}}^{l-1}\right), \end{array}$$

where *x*_*k*_^*l*^ represents the output of the *k*th neuron of layer *l*, subsample represents the subsampling operation, and *x*_*k*_*cluster*__^*l*−1^ represents the *k*th output cluster of layer *l* − 1.

The input and output structures of the main modules of the proposed model are shown in Table 2. The size of the convolution kernel of the first convolution layer is 9, and the number of convolution kernels is 32. In the following 6 feature extraction modules, the convolution kernel of the convolution layer in each feature extraction module is 3∗1, and the number of convolution kernels is 64, 64, 128, 128, 256, and 256, respectively. The filter of all the pooling layers used in the method is 2∗1, and the step size is 2. The method of using multiple small convolution kernels instead of a single large convolution kernel is used to set network parameters, and the network designed with this idea obtains a better classification effect [27, 28].

#### 2.3.3. Description of the GRU Module

As shown in Figure 3, the features extracted by CNN are input to the GRU layer. From the structure of CNN in equation (1), the sample processing of ordinary CNN is calculated independently at every moment. It pays more attention to the spatial correlation of features, which makes it difficult to extract all the features of the time series only by using the CNN structure [29]. From the internal structure of GRU shown in Figure 4, the output of each neuron layer in GRU affects the output at subsequent moments, so it can be used to describe time series and solve the problems of gradient disappearance and gradient explosion in long sequence training [30, 31]. Also, note that the GRU uses two gating units to determine how the new information is combined with the previous information and how much of the previous information is retained to calculate the new state, which greatly saves computation in the time feature extraction process. Equations (3), (4), (5), and (6) are the state of the cell in Figure 4 and the output of each layer at every moment:

(3) $$\begin{array}{c} r_{t}=\sigma \left(W_{xr}^{T}\cdot x_{t}+W_{\text{or}}^{T}\cdot o_{t-1}+b_{r}\right), \end{array}$$

(4) $$\begin{array}{c} z_{t}=\sigma \left(W_{xz}^{T}\cdot x_{t}+W_{oz}^{T}\cdot o_{t-1}+b_{z}\right), \end{array}$$

(5) $$\begin{array}{c} {\tilde{o}}_{t}=\tanh\left(W_{x\tilde{o}}^{T}\cdot x_{t}+W_{o\tilde{o}}^{T}\cdot \left(r_{t}⊗o_{t-1}\right)+b_{\tilde{o}}\right), \end{array}$$

(6) $$\begin{array}{c} o_{t}=z_{t}⊗o_{t-1}+\left(1-z_{t}\right)⊗{\tilde{o}}_{t}, \end{array}$$

where $W_{xr},W_{xz},W_{x\tilde{o}}$ represents the weight matrix of the corresponding vector, $W_{\text{or}},W_{oz},W_{o\tilde{o}}$ represents the weight matrix of the previous moment, and $b_{r},b_{z},b_{\tilde{o}}$ represents the deviation.

### 2.4. Architecture of Proposed Model

The selection of loss function and optimizer is as important to the accuracy as the construction of a network structure [32]. This section describes the optimizer and loss function in the proposed method.

#### 2.4.1. Cost Function

The loss function is used in model training to show the gap between the predicted effect and the actual data. The smaller the loss function is in the training process, the more accurate the classification effect of the model will be. The cross-entropy function is selected as the cost function in this work, which can overcome the shortcoming of slow parameter updates of the traditional loss function [33]. Equation (7) shows its principle:

(7) $$\begin{array}{c} J=-\frac{1}{N}\left[y_{n}\log\left({\hat{y}}_{n}\right)+\left(1-y_{n}\right)\log\left(1-{\hat{y}}_{n}\right)\right], \end{array}$$

where *J* is the total cost, *N* is the number of training data, *y*_*n*_ is the expected output, and ${\hat{y}}_{n}$ is the actual output generated by the network.

#### 2.4.2. The Optimizer

In 2014, Kingma and Leiba proposed the Adam optimizer, which combines the advantages of Adagrad and Rmsprop and calculates the update step size by using gradient first-order moment estimation and second-order moment estimation [34]. The Adam optimizer can automatically adjust the learning rate with a small amount of computation, and usually, there is no need to adjust the learning rate; it is well suited to the datasets with large samples [35, 36].

## 3. Results

In this section, the training method of the model is introduced first. Then, the experimental results were mainly studied, and the effects of each step of the experiment on the classification performance were compared.

### 3.1. Setup

The dataset is randomly divided into the training set and test set in the order of 8 : 2. The training set is input into the proposed network to train the classification model, and the classification effect of the test set is used to evaluate the performance of the model.

The proposed network is implemented using the Keras framework, and the convolutional neural network is coded using Python. The experiment was set up on an Intel Core i5-9600@3.10 GHz CPU; the GPU was Radeon520. The trained model is stored in the HDF5 file.

### 3.2. Evaluation

To evaluate the effectiveness of the model, accuracy, sensitivity, and F1-score were used to evaluate the model performance. Accuracy is the most common standard for evaluating model performance, representing the proportion of correctly predicted samples to the total samples. Precision reflects the proportion of true positive examples judged as positive examples by the classifier. Sensitivity represents the proportion of correctly classified true positive samples to all true positive samples. F1-score (balanced average) is the calculation result of integrating model sensitivity and precision, and its value is more inclined to the index with a smaller value. Definitions of accuracy, sensitivity, and F1-score are shown in formula (8), (9), (10), and (11):

(8) $$\begin{array}{c} \text{accuracy}=\frac{\text{TP}+\text{TN}}{\left(\text{TP}+\text{TN}\right)+\left(\text{FP}+\text{FN}\right)}, \end{array}$$

(9) $$\begin{array}{c} \text{sensitivity}=\text{recall}=\frac{\text{TP}}{\text{TP}+\text{FN}}, \end{array}$$

(10) $$\begin{array}{c} \text{precision}=\frac{\text{TP}}{\text{TP}+\text{FP}}, \end{array}$$

(11) $$\begin{array}{c} \text{F}1‐\text{score}=\frac{2\text{precision}\cdot \text{recall}}{\text{precision}+\text{recall}}, \end{array}$$

where *TP* represents the number of true positive samples, *TN* represents the number of true negative samples, *FP* represents the number of false positive samples, and *FN* represents the number of false negative samples.

### 3.3. Experiment

Different structures of CNN have different feature extraction capabilities. With the deepening of the convolutional layer, the classification performance of the CNN classifier will become stronger. However, when the convolutional layer deepens to a certain threshold, the performance of the classifier is no longer strong, and the training time will be longer. It should also be noted that the mapping relationship between the heartbeat category and its waveform is very complex, and the LFEM of the double-convolutional structure has higher accuracy than the feature extraction module of the single convolutional layer. To find the most suitable classification model, 10 kinds of CNN structures were used for evaluation on the MIT-BIH database.  Table 3 shows the classification accuracy of each structure, D1-D5 represent the classification results of CNN built by 2, 4, 6, 8, and 10 LFEMs, and S1-S5 represent the classification results of CNN built by 2, 4, 6, 8, and 10 convolutional layers. Due to the data length limitation, we remove the pooling layer of the seventh and eighth feature extraction modules, respectively, in the two 10-layer convolution structures. Among these ten convolutional structures, the number of convolutional kernels at 1-10 layers is 64, 64, 128, 128, 256, 256, 256, 256, 256, and 256, respectively. The size of the convolutional kernels is 3∗1, and the step size is 1. The filters for all pooling layers used in this method are 2∗1, and the step size is 2.

As can be seen from Table 3, for the CNN classifier with the same number of layers, the classifier with LFEM is generally better than the classifier stacked with a single convolutional layer. It can also be seen from Table 3 that when the depth of the CNN model with LFEM reaches 6 layers, deepening the number of network layers cannot further improve the classification performance of the model. This indicates that the number of neural network layers in the D3 structure can best extract features from the MIT-BIH database. Therefore, D3 was chosen as the final CNN structure.

The data enhancement technology and GRU were added to the proposed method. As can be seen from Figure 5, the model has a significantly better ability to classify S and F beats with a small number of beats after the use of the data enhancement technology.

The confusion matrix obtained by using the proposed method for MIT-BIH arrhythmia database classification is shown in Figure 6. It can be seen from the confusion matrix that the overall performance of the proposed method is very good. Observe the diagonal value of the matrix, and it shows that the correct sample proportion reaches more than 99%.  Figure 7 shows the receiver operating characteristic (ROC) curve for the proposed model, the diagonal is a random classification model of the ROC curve, and the ROC curve to the left upper corner of the near axis represents better results [37]. The Area Under Curve (AUC) represents the size of the area under the ROC curve, and it represents the probability that a positive example is predicted to be ahead of a negative example [38]. As can be seen from Figure 7, the AUC of the proposed ECG detection method is close to 1.

The training accuracy and loss curves obtained when 200 epochs were trained by this method are shown in Figures 8 and 9. The accuracy curve is observed, and the training accuracy and testing accuracy of the model are stable at more than 99% after 130 epochs, indicating that the model has a good classification effect on the MIT-BIH database. The precision curve and the loss function curve of the whole training process are relatively stable, and the loss function is stable between 0 and 0.2; it shows that the cross-entropy function has good performance.

To evaluate the performance of the CNN-GRU model, a CNN-LSTM model that only changes GRU to the LSTM structure is compared with the proposed model. The detailed information of the classification performance of CNN-GRU and CNN-LSTM models is shown in Table 4. The accuracy, sensitivity, and F1-score of the CNN-LSTM model reached 99.02%, 99.05%, and 98.87%, and the accuracy, sensitivity, and F1-score of the CNN-GRU model was 99.61%, 99.33%, and 99.42%, respectively. After summarizing Table 4, it can be seen that the overall performance of the CNN-GRU network is better than that of the CNN-LSTM network.

### 3.4. Compare the Proposed Method with Other Existing Methods

Table 5 provides a comparative analysis of the existing and proposed methods. Four state-of-the-art models were used to classify the MIT-BIH database and compare the accuracy, sensitivity, and F1-score with the proposed network. Compared with the proposed network whose performance is more than 99% in accuracy and sensitivity, Jun et al.'s [10], Acharya et al.'s [11], Hannun et al.'s [12], and Ihsanto et al.'s [13] models had much lower accuracy, sensitivity, and F1-score. This is due to the use of effective denoising and data segmentation technology in the preprocessing stage and a reasonable method in the design of the network; the use of a local feature extraction module of the double-convolutional structure is also an important reason to achieve excellent results.

## 4. Discussion

In this paper, a new classification method based on the characteristics of ECG signals is proposed. Firstly, the noise and artifacts in the signals are removed through wavelet decomposition and reconstruction, and the data enhancement technology is designed to expand the dataset. Then, the dual convolution structure is used to construct the local feature extraction module, and the CNN structure which can better extract the characteristics of complex ECG signals is designed. Finally, GRU is introduced in combination with CNN to help the classifier obtain the ability to extract the time dependence when classifying ECG sequences, which can improve the classification performance of the classifier. The total classification accuracy of the model in the MIT-BIH database can reach 99.61%, the average sensitivity and F1-score can reach 99.33% and 99.42%, and the experiments show that the model has a strong learning ability. In addition, compared with Hannun et al.'s method, the proposed method achieves a better classification effect with a shallower network. The proposed network can also be applied to other one-dimensional signals.

## Figures and Tables

**Figure 1:** Signal before and after denoising comparison. There is a noise interference signal in the original signal, and this process reduces the influence of the noise signal on the classification process.

**Figure 2:** The architecture of the proposed model.

**Figure 3:** GRU model.

**Figure 4:** The internal structure of GRU.

**Figure 5:** The proposed data enhancement technique and the influence of GRU on sensitivity.

**Figure 6:** Confusion matrix for the proposed model.

**Figure 7:** The ROC of the proposed model.

**Figure 8:** Accuracy curve of ECG classification.

**Figure 9:** Loss curve of ECG classification.

**Table 1:** Summary of the heartbeats. Reproduced with permission from Rajesh and Dhuli [14].

The AAMI heartbeat class description	Annotations of MIT-BIH heartbeats
Nonectopic beats (N)	Normal beats
	Left bundle branch block beats
	Right bundle branch block beats
	Nodal (junctional) escape beats
	Atrial escape beats
Supraventricular ectopic beats (S)	Aberrated atrial premature beats
	Supraventricular premature beats
	Atrial premature contraction
	Nodal (junctional) premature beats
Ventricular ectopic beats (V)	Ventricular flutter wave
	Ventricular escape beats
	Premature ventricular contraction
Fusion beats (F)	Fusion of ventricular and normal
	Beats
Unknown beats (Q)	Paced beats
	Unclassifiable beats
	Fusion of paced and normal beats

**Table 2:** The output shape of the main module.

The name of the module	Output
Input	186∗1
Conv	186∗32
LFEM1	93∗64
LFEM2	47∗64
LFEM3	24∗128
LFEM4	12∗128
LFEM5	6∗256
LFEM6	3∗256
Reshape	1∗768
GRU	1∗768
Dense	96
Softmax	5

**Table 3:** Comparison of accuracy of different CNN structures.

The types of CNN structures	D1	D2	D3	D4	D5	S1	S2	S3	S4	S5
Average accuracy after 10 training sessions (%)	96.33	97.45	98.84	98.73	98.78	94.99	95.78	96.73	97.21	97.15

**Table 4:** Accuracy comparison between CNN-LSTM and CNN-GRU.

Classifier	Accuracy (%)	Sensitivity (%)	F1-score (%)
CNN-LSTM	99.02	99.05	98.87
CNN-GRU	99.61	99.33	99.42

**Table 5:** Comparison of the proposed network and state-of-the-art methods.

Work	Accuracy (%)	Sensitivity (%)	F1-score (%)
Jun et al. [10]	97.55	97.05	97.44
Acharya et al. [11]	93.50	93.35	93.41
Hannun et al. [12]	94.95	95.46	94.91
Ihsanto et al. [13]	99.02	76.32	80.97
Proposed model	99.61	99.33	99.42

## Data Availability

The MIT-BIH arrhythmia database used to support the findings of this study can be obtained from the following connection: https://physionet.org/content/mitdb/1.0.0/.
